# CT Image Features Based on the Reconstruction Algorithm for Continuous Blood Purification Combined with Nursing Intervention in the Treatment of Severe Acute Pancreatitis

**DOI:** 10.1155/2022/2622316

**Published:** 2022-03-28

**Authors:** Yanyan Liu, Mingli Gu, Liping Liu, Lunmeng Cui, Aimin Xing

**Affiliations:** Department of Critical Care Medicine, Affiliated Hongqi Hospital of Mudanjiang Medical University, Mudanjiang 157011, Heilongjiang, China

## Abstract

The aim of the study was to explore the CT images of the iterative reconstruction algorithm to evaluate the curative effect of continuous blood purification combined with nursing intervention in the treatment of severe acute pancreatitis (SAP). A total of 100 patients with SAP treated by the bedside continuous venous hemofiltration purification method in a hospital were selected. The control group (*n* = 50) was given a routine treatment, and the observation group (*n* = 50) was treated with the continuous blood filtration mode for blood purification based on the routine treatment. In the CT image scanning of periodontitis patients, the iterative reconstruction algorithm was introduced to reduce image noise, and the CT values under the algorithm were statistically analyzed. The results showed that IL-1, IL-6, and IL-8 after treatment were significantly lower than those before treatment (*P* < 0.05). The symptoms effectively improved with continuous blood purification combined with nursing intervention in patients with SAP. After the use of the iterative reconstruction algorithm, the image quality, image information, and image MSE significantly improved. The image noise with 50% dose reduction was the lowest, but the reconstruction algorithm improved the low contrast resolution (*P* < 0.05). CT images based on the reconstruction algorithm can clearly display the lesion characteristics of the patients, and the reconstruction algorithm is feasible to improve the spatial resolution of CT images.

## 1. Introduction 

Acute pancreatitis (AP) is one of the common clinical abdomen pains with high mortality. The mortality rate of severe acute pancreatitis (SAP) in China is 25%–40%, and that in foreign countries is 15%–30%, mainly due to secondary infection caused by pancreatic and surrounding tissues [1]. The clinical manifestations of SAP are pancreatic edema, hemorrhage and necrosis, and systemic inflammatory response. SAP is one of the common critical illnesses in the emergency department. Active inflammatory factors in the body during the onset lead to the release of a large number of cytokines, leading to the aggravation of the disease [2]. The secondary infection of the pancreas and the peripancreatic tissue further develops into multiple organ failure, which seriously threatens the life of patients and produces a higher mortality [3]. At present, the effective treatment for SAP is mainly the continuous blood purification treatment, which can quickly purify the toxins in patients, so as to reduce the impact of the toxins on the bodies of these patients, and the inflammatory symptoms disappear [4]. SAP has a variety of causes. Excessive drinking and drinking can cause poor drainage of the pancreatic duct, increased pressure in the pancreatic and biliary systems, and a high concentration of protease excretion disorders, resulting in the rupture of pancreatic vesicles. Bile duct inflammation, stones, edema, and other lesions can cause ampulla obstruction, bile reflux into the pancreatic duct, and trypsinogen activation. In clinical practice, many infectious infections can also promote the occurrence of acute pancreatitis [5, 6]. Continuous blood purification is a new blood purification method that continuously and slowly removes the water and solute in patients. By inputting a large amount of replacement solution to the patients and giving them intravenous nutritional support, it can promote the recovery of the patient's condition, and has a good effect in severe cases[7, 8].

CT has been continuously applied in clinical diagnosis, and has proven to be an important method for the diagnosis of many diseases. In many cases, X-rays cannot provide sufficient information on the actual size of the lesion and the spatial position of the anatomical landmarks [9, 10]. CT scanning can show the volume increase of diffuse pancreas and the distribution of the pancreatic density, and enhanced scanning shows the pancreas has uneven mild enhancement, which can accurately observe the lesion site. Detecting acute pancreatitis using CT has advantages such as: fast CT scanning speed, strong ability of multiplanar reorganization and grading ability, avoiding respiratory movement artifacts and gastrointestinal gas influence, with high sensitivity and specificity. The severity of pancreatitis and the involvement of adjacent organs can be clearly judged, and the CT severity index score can be performed. However, in terms of the actual situation, the CT scan range is limited, and the scanned part is large, which leads to the detection data being truncated and not comprehensive. This situation will cause the possibility of inaccurate inspection results in the reconstruction of CT images. Moreover, due to the limitation of angles, CT images will produce a large number of artifacts in the scanning process. At present, how to reduce the generation of image artifacts in the case of reducing the radiation during CT examination has become a major research hotspot in the field of imaging examination.

With the development of algorithm technology, the iterative reconstruction algorithm has been widely studied and applied in CT images. It belongs to a new infrared imaging technology, and the conditions required for scanning imaging are relatively low. In the case of large calculation cost, the iterative reconstruction algorithm is still a good reconstruction method for projection data with incomplete information or noise [11–13]. CT image reconstruction is based on many mathematical and physical operations. Its purpose is to reduce image noise and improve image resolution. Therefore, it is very important to reasonably use the reconstruction algorithm and maximize the effect of the algorithm [14–16].

In summary, the data of CT images using the iterative reconstruction algorithm are reconstructed and applied in the diagnosis of GC diseases to improve the accuracy of the diagnosis, and reasonable analysis is carried out through research. It is hoped that CT images based on the reconstruction algorithm can clearly present the lesions of the patients, improve the detection method, and provide reference for the diagnosis of diseases in clinic settings.

## 2. Methods

### 2.1. General Information

One hundred patients with SAP treated in a hospital from January 2019 to December 2020 were randomly divided into an observation group and a control group. In the control group, there were 26 males and 24 females, aged 29–50 years, with an average age of (41.54 ± 2.18) years, including 32 patients with hypertension and 18 patients with simple periodontitis. There were 20 males and 30 females in the observation group, aged 28–52 years old, with an average age of (43.54 ± 2.76) years. There were 22 patients with hypertension and 28 patients with simple periodontitis. The causes of SAP in the two groups were biliary pancreatitis, hyperlipidemia, overeating, and excessive alcohol consumption. There was no significant difference in the general data of the patients (*P* > 0.05), indicating comparability. This study had been approved by the Ethics Committee of hospital and all patients signed the informed consent form.

Inclusion criteria: (1) Patients who conform to the diagnostic criteria of acute severe pancreatitis. (2) Patients voluntarily participated in the study. (3) Patients without immune system diseases or infectious diseases. Exclusion criteria: (1) Incomplete clinical data. (2) Patients who are unwilling participants. (3) Patients with mental illness.

### 2.2. Method

The control group was treated with conventional treatment, fasting, and continuous gastrointestinal decompression. Painkillers and antispasmodics could be selected to correct the water, electrolyte, and acid–base balance of the patients. Infected patients were treated with anti-infective drugs. If there were shock patients, shock drugs could be used and enteral and parenteral nutrition could be given to patients reasonably. The vital signs of the patients were comprehensively tested.

On the basis of the conventional treatment, the observation group was treated with the continuous blood filtration mode for blood purification. Cardiopulmonary bypass was established in the right femoral vein intubation of the patient, and continuous blood filtration was performed. The flow rate of the replacement solution was determined according to the patient, and 1500–2000 ml/h was located. The replacement solution formula was flexibly and reasonably formulated in combination with the electrolyte disorder and acid–base balance of the patient, and the dosage of sodium bicarbonate, calcium, and potassium in the replacement solution was personalized and adjusted. The blood flow was 150–200 ml/h, which could be adjusted according to the patient's capacity state. The purification time was 24 h, and the vital signs of the patients were closely monitored. If biochemical indexes were obviously normal, symptoms were significantly alleviated, and if serum amylase decreased, the blood purification treatment could be stopped. Continuous purification once a day or every other day according to the patient's condition, the cumulative treatment time was more than 72 hours.

Patients were examined by Dual source computed tomography. The examination process was described in detail to the patients before scanning. The patients were in supine position, and the peripheral venous pathway of the lower limb (any lower limb) was established to connect the ECG and the blood oxygen monitor. Before the examination, the patients were sedated by professional anesthesiologists. The dosage of the anesthetic was 2 mL/kg, and the duration was 10–15 minutes. In addition, the ECG, respiration, and peripheral blood oxygen saturation of the patients were monitored. The obtained CT images were transmitted to the workstation and processed by Functool II software. Post-processing workstation: Vitrea3.9 version post-processing workstation.

Firstly, the ECG gating technology was used. The tube voltage was 80 KV, and the tube current parameters were adjusted according to body weight. The machine automatically gave pitch, and the periodic exposure was automatic. The Ultravist (370 mg/mL) was used as the contrast agent, and the flow rate of the MEDRED double-tube high-pressure syringe was 0.12 mL/s/kg. After intravenous injection (the injection time was 20 seconds), the saline was injected at the same flow rate for 10 seconds. The range was then selected for scanning.

### 2.3. Observation Indicators

For the determination of inflammatory factors, 5 mL blood was collected on an empty stomach without anticoagulation, separated at 3, 000 r/min for 10 min, and stored at −20°C for later use. IL-6, IL-8, and IL-1 were determined by double-antibody Sandwich ELISA in Roche automatic chemiluminescence analyzer. Measurements were strictly in accordance with instructions.

PACHE II score: The physical condition of the patients was scored 72 hours before and after treatment. The higher the score, the more serious the disease. The score included chronic health status, age, and acute physiology score, with the highest score of 71 points.

The evaluation index of the algorithm was the mean square error (MSE).

(1) $$\begin{array}{c} \text{MSE}=\frac{1}{M}{\sum_{\text{i}=1}^{M}\left(yi-\hat{y}i\right)}^{2}. \end{array}$$

### 2.4. CT System Imaging Flow Chart

The imaging of CT is similar to X-rays. The X-ray passes through different tissues of the human body, and has different gray levels on CT images. After X-ray penetration, the corresponding attenuation of different tissues and organs is also different. X-ray projection data are the most primitive image information data. The CT image uses a highly collimated X-ray to scan a certain thickness of the patient's body. The detector records the attenuation information of the X-ray during the scanning process.  Figure 1 shows the imaging flow chart of the CT system. The converter converts the analog information into digital information, and then enters the electronic calculation. The information flow is provided by the high-voltage generator to generate X-rays. The CT machine is also rotated at this time. The detector collects data continuously. According to the scanning of the patient's body, it is converted into electrical signals. The DAS system is converted into digital electrical signals. The slip ring system is used to reconstruct the image.

### 2.5. Improvement of Image Noise by the Iterative Reconstruction Algorithm

The complete CT iteration is called full iterative reconstruction, including back projection and front projection. The connection of these two parts is also mainly completed by the iterative method. The working principle of the iterative algorithm is to reduce the noise in the front and rear projection domains. At the beginning of each calculation, image assumptions should be made, i.e., a similar initial value for each image is set, and then the possible projection value is calculated after the light passes through the human body. Firstly, a virtual image is constructed, and the iterative model is constructed including the construction of the noise model. According to the actual measurement value, the hypothetical image is continuously modified repeatedly. The calculation results and the real projection results are analyzed to obtain the corresponding correction results. The pixel value can be corrected many times until all the images are completed. The purpose of iterative reconstruction is to obtain a more realistic original image. The CT iterative image includes two parts: the front projection and the back projection. The principle of signal-to-noise ratio reduction is shown in Figure 2. The image is assumed, and then the initial value is set. The projection value of the light passing through the human body is calculated. The correction results show that the signal-to-noise ratio of the image is reduced, and the reconstructed image is obtained. The iterative reconstruction image is closer to the real image, and CT image reconstruction for patients can greatly reduce the scanning dose and effectively improve the image quality. The yellow arrow indicated the location of the lesion in Figure 2.

### 2.6. Application Principle

It is supposed that the size of the CT image is *h∗w*, and the projection process can be expressed as follows:

(2) $$\begin{array}{c} U^{YX}=E^{YX\times hw}•R^{hw^{1}}. \end{array}$$

*R*^*hw*^1^^ represents the image with size vector as *hw*^1^; *E*^*YX*×*hw*^ represents the projection coefficient with matrix as *YX* × *hw*; *Y* means the maximum projection value obtained at different angles, and *X* means different angles; *U*^*YX*^ is the projection vector with a size of *YX*.

The expression after image reconstruction is as below:

(3) $$\begin{array}{c} B^{hw*}=E^{YX\times hw*}•U^{YX}. \end{array}$$

*B*^*hw∗*^ denotes the image with size *hw*^1^; *E*^*YX*×*hw∗*^ represents the generalized inverse of the projection coefficient as *E*^*YX*×*hw*^. However, due to the complexity and time-consuming nature of the *E*^*YX*×*hw∗*^ calculation process, it needs to be improved. Therefore, it is replaced by another calculation method to save time.

Based on the following calculation principles, the first-order iterative method is used to obtain *E*^*∗*^.

When the *E*^*YX*×*hw∗*^ initial estimation is *P*_0_ and the residual is *C*_0_=*U*_*R*(*T*)_^*YX*^ − *E*^*YX*×*hw*^•*P*_0_, *γC*_0_ < 1 and *C*_0_ represents the radius of the spectrum; *U*_*R*(*T*)_^*YX*^ means the *E*^*YX*×*hw*^ orthogonal matrix. According to the above contents, the sequence {*P*_0_, *P*_1_,…*P*_*K*_,  *P*_*K*+1_,…} can be expressed as follows:

(4) $$\begin{array}{c} \left\{\begin{array}{c} P_{K+1}=P_{K}+P_{0}-P_{0}•E^{YX\times hw}•P_{K}\\ K=0,1,\ldots \end{array}\right). \end{array}$$

When *K*⟶*∞*, the upper convergence *E*^*YX*×*hw∗*^ is obtained, and the corresponding residual sequence can be expressed as

(5) $$\begin{array}{c} \left\{\begin{array}{c} \left\|C_{K+1}\right\|\leq \left\|C_{0}•C_{K}\right\|\\ K=0,1,\ldots \end{array}\right). \end{array}$$

The norm multiplication calculation of the matrix conforms to the following equation (6).

(6) $$\begin{array}{c} \left\|C_{K}\right\|=U_{R\left(T\right)}^{YX}-E^{YX\times hw}•P_{K}. \end{array}$$

In order to make the calculation simpler, the *E*^*YX*×*hw∗*^ approximation can be set as follows:

(7) $$\begin{array}{c} P_{0}=\theta E^{YX\times hw*•t}. \end{array}$$

*E*^*YX*×*hw∗*•*t*^ means a transposition of *E*^*YX*×*hw*^; *θ* represents a real value, consistent with *θE*^*YX*×*hw∗*•*t*^.

(8) $$\begin{array}{c} \theta \in \left(0,\frac{2}{\lambda_{1}E^{YX\times hw}}•E^{YX\times hw•t}\right). \end{array}$$

*λ*_1_*E*^*YX*×*hw*^•*E*^*YX*×*hw*•^ expresses the maximum non-zero eigenvalue of *E*^*YX*×*hw*^•*E*^*YX*×*hw*•^.

In order to reduce the difficulties in calculating *E*^*YX*×*hw*^ and *E*^*YX*×*hw*•*q*^, the projection vector *U*^*YX*^ is added to both sides of equation (4) in the form of multiplication, and equation (9) can be obtained.

(9) $$\begin{array}{c} \left\{\begin{array}{c} P_{K+1}U^{YX}=P_{K}U^{YX}+P_{0}U^{YX}-P_{0}•E^{YX\times hw}•P_{K}•U^{YX}\\ K=0,1,\ldots \end{array}\right). \end{array}$$

*P*_*K*+1_*U*^*YX*^ is the *K*+1 reconstructed image *R*_*K*+1_^*i*^; *N*_*K*_•*U*^*YX*^ represents the *K* reconstructed image *R*_*K*_^*i*^; *P*_0_•*U*^*YX*^ denotes the original image *R*_0_^*i*^; *P*_0_•*E*^*YX*×*hw*^•*P*_*K*_•*U*^*YX*^ denotes the projection of the image *R*^*i*^, and then the image is reconstructed. The reconstruction times *θ* of *P*_0_•*E*^*YX*×*hw*^•*P*_*K*_•*U*^*YX*^ are replaced with the FBP algorithm.

If *hw* < *YX*, *θ*=1; if *PP* < *YX*, *θ* < 2^−(*hw* ÷ *YX*)^.

In order to evaluate the application effect of the algorithm, the following experiments are carried out. It is supposed that the *θ* value is 1.

The schematic diagram of the iterative reconstruction algorithm is illustrated in Figure 3.

### 2.7. Application Steps

The application steps of the iterative reconstruction algorithm are as follows:

**Step 1 .**

*θ* is initialized and the condition *φ* is terminated.

**Step 2 .**

In the case of *K*=0, the FBP algorithm is adopted to preprocess the original image, and *R*_*fbp*_^*i*^*R*_0_^*i*^=*θR*_*flp*_^*i*^ is obtained.

**Step 3 .**

*R*_*K*_^*i*^ is projected to get the projection value *U*^*YX*^ _*K*_.

**Step 4 .**

The reconstructed image combining *U*^*YX*^ _*K*_ with the FBP algorithm is multiplied with *θ* to obtain *R*_*r*_.

**Step 5 .**

The reconstructed image is corrected, and *R*_*K*+1_^*i*^=*R*_*K*_^*i*^+*R*_0_^*i*^ − *R*_*r*_^*i*^.

**Step 6 .**

Δ=‖*R*_*K*+1_^*i*^ − *R*_*K*_^*i*^‖, and $\left\{\begin{array}{c} \left\|R_{K+1}^{i}-R_{K}^{i}\right\|\leq K\\ K=k+1 \end{array}\right)$.

**Step 7 .**

If Δ > *φ*, Step 3 is performed, conversely, end of calculation (Figure 4).

### 2.8. Statistical Analysis

Relevant data of chronic periodontitis patients were recorded by SPASS 21.0 statistical software. The measurement data were expressed as ($\bar{\text{x}}$ ± *s*), and the *t*-test was used. The count data were expressed as (*n*, %), and *P* < 0.05, i.e., the difference was statistically significant.

## 3. Results

### 3.1. General Data

Table 1 shows the general data of the two groups of patients. There was no significant difference between the patients (*P* > 0.05). In the control group, the average age was (41.54 ± 2.18) years, including 8 cases of biliary pancreatitis, 11 cases of hyperlipidemia, 22 cases of overeating, and 9 cases of alcoholics. The average age of the patients in the observation group was (43.54 ± 2.76) years, including 10 cases of biliary pancreatitis, 9 cases of hyperlipidemia, 19 cases of overeating, and 12 cases of alcoholics.

### 3.2. CT Images

When the same dose was used in Figure 5, from the CT image, there was exudation around the pancreas, a small amount of effusion, and scattered cellular inflammatory changes. Figure C showed peripancreatic exudation in a case of simple pancreatitis. No obvious necrotic area was observed.

### 3.3. Iterative Algorithm CT Image Reconstruction

Iterative reconstruction algorithm is based on the estimation of the statistical model of observation data. The CT images of a patient with severe pancreatitis complicated with necrosis are shown in Figures 6(a) and 6(b). The secondary pancreatic abscess is formed on the basis of necrosis. There were obvious necrotic liquefaction foci in the abscess area, and the necrotic area was in the red box. The red arrow indicated the location of the lesion.  Figure 6(c) shows the formation of pseudocysts around the spleen in the patients. Circular nodules in the red frame can be seen in the pseudocysts on the splenic hilum side, showing a significant enhancement similar to the large blood vessels in the abdominal cavity, which is the manifestation of pseudoaneurysm.

### 3.4. Comparison of the Reconstruction Algorithm Image Results

In CT imaging, the noise of the image decreases after applying the iterative reconstruction algorithm (Figure 7). With the reduction of the use dose, the spatial resolution of the image is effectively improved. The image noise with 50% dose reduction is the lowest (Figure 8), but the reconstruction algorithm improves the low-contrast resolution.

### 3.5. MSE of the Iterative Reconstruction Algorithm CT Images

The iterative reconstruction algorithm can restore the original image after a certain number of iterations (Figure 9). The MSE is closer to zero, and the representation effect is better. The image quality is better after the reconstruction algorithm.

### 3.6. Comparison of the Reconstructed Images

The simulation of low-dose CT image reconstruction was used. The template was 128 × 128 mm. The algorithm operating system was Window 10 32 bit SPI. The processor was Intelku 2 dual-core T6400@2.00 GHz processor, and the inner was 2G. The reconstruction image comparison shown in Figure 10(a) was an ideal projection domain image and was relatively clear.  Figure 10(b) contained the noise projection domain image, and the particle sense was obvious.

### 3.7. APACHE II Score of the Two Groups

From Figure 11, the APACHE II scores of the two groups were decreased after treatment, indicating that the conditions of the two groups improved. After treatment, the difference between the observation group and the control group was significant (*P* < 0.01), indicating that the observation group showed better curative effect.

### 3.8. Comparison of the Survival Rate between the Two Groups

From Table 2, there were five deaths in the control group, of which two died of renal failure, one died of infective shock, and two died of fungal sepsis. One patient died of multiple organ failure in the observation group. The survival rate of the observation group was significantly higher than that of the control group (*P* < 0.01).

### 3.9. Comparison of the Two Groups of Patients with Severe Factor Levels

As shown in Figure 12, the levels of inflammatory factors in the two groups were compared and analyzed. After treatment, the levels of the inflammatory factors were significantly decreased compared with those before treatment, and the levels of IL-1, IL-6, and IL-8 after treatment were significantly lower than those before treatment (*P* < 0.05), indicating that both treatments could improve the symptoms of the patients.

## 4. Discussion

Continuous blood purification is a new blood purification treatment method, which can continuously and slowly remove the solute and water in the blood, improve the patient's immune system, and maintain the stability of the internal environment. Continuous blood purification treatment uses the strong adsorption of polymer material filter to remove IL-6, IL-1, IL-8 inflammatory factors and toxic metabolites during tissue injury, which can promote the recovery of organ function and regulate immune function [17–19]. Zhu et al. [20] found that continuous blood purification can rapidly reduce the blood amylase and lipase in children with SAP, help maintain the stability of the internal environment, block the systemic inflammatory response, improve organ function, and maintain fluid balance. In this study, the inflammatory factors of IL-6, IL-1, and IL-8 in the two groups reduced after treatment. Continuous blood purification can effectively improve patients with SAP.

As a fast-scanning technology, CT three-dimensional imaging can not only reduce the time of operation and imaging in the detection process, but also obtain more CT images and data information of lesions under the same scanning condition. Then, with the assistance of computers, more high-quality CT images are obtained for the diagnosis of patients' diseases. The processed CT images can not only be as intuitive as endoscopic images, but also improve the detection rate of small lesions. On this basis, further reconstruction of CT images by the iterative algorithm can improve the image quality. The iterative algorithm divides the whole image processing process into many times and gradually improves the image processing. During most low-dose scanning, the scanned image processing parameters must be optimized to maximize the image quality. The algorithm and various noise reduction technologies can smooth the image. It is found that the iterative reconstruction algorithm effectively optimizes the CT image quality, information quantity, and mean square error. Among them, the MSE is the optimal value with the result close to 0. The iterative algorithm was used to reconstruct and denoise CT images. The results showed that the image quality, image information, and image MSE significantly improved after the use of the iterative reconstruction algorithm. The CT image based on the reconstruction algorithm could clearly display the lesion characteristics of the patients, and the reconstruction algorithm was feasible to improve the spatial resolution of the CT images. Tirkes [21] stated in the literature that CT and MRI cholangiopancreatography are common cross-sectional imaging studies for the evaluation of chronic pancreatitis. The reconstruction algorithm is applied to CT three-dimensional imaging. With the reduction of the dose, the image spatial resolution is effectively improved. Comparing the image noise, it is found that the image noise with 50% dose reduction is the lowest, and the reconstruction algorithm can improve the low-contrast resolution. Gupta et al. [22] used CT to scan the gastrointestinal tract of patients with acute pancreatitis, and found CT features such as maximum thickness of the intestinal wall, extrapancreatic necrosis, and intestinal wall thickening. CT is helpful to predict gastrointestinal fistula in patients with acute pancreatitis. Abdullah et al. [23] applied the iterative reconstruction algorithm to CT angiography. The results show that the iterative reconstruction algorithm can effectively reduce the noise of CT images and improve the signal-to-noise ratio. The results show that the iterative reconstruction algorithm has a good-quality effect in the CT image scanning of SAP patients.

## 5. Conclusion

After the optimization of the iterative reconstruction algorithm, the quality of the CT image improved and the signal-to-noise ratio effectively improved. The reconstructed image algorithm can improve the quality of low-dose CT reconstructed images. This algorithm is feasible in the CT image application. The effect of continuous blood purification nursing intervention in the treatment of SAP patients is better than that of the ordinary routine treatment. There are many limitations, and the number of iterations of the algorithm is not repeated enough. In the future, the accuracy of the algorithm can be discussed from the number of iterations. Low-dose CT imaging is a research subject with a wide range. Compared with the actual situation, there must be differences in the simulated noise of low-dose CT. How to eliminate these differences can be studied in the next step.

## Figures and Tables

**Figure 1:** Flow chart of the CT system imaging.

**Figure 2:** Process diagram of the iterative reconstruction algorithm.

**Figure 3:** Schematic diagram of the iterative reconstruction algorithm.

**Figure 4:** Flowchart of algorithm steps.

**Figure 5:** CT images of acute pancreatitis (patient with acute simple pancreatitis, female, 57 years old).

**Figure 6:** Three-dimensional CT images of patients with SAP. (a, b) The CT images of a patient with severe pancreatitis complicated with necrosis. (c) The formation of pseudocysts around the spleen in the patients.

**Figure 7:** Image quality assessment of the iterative reconstruction algorithm.

**Figure 8:** Improvement of signal to noise ratio.

**Figure 9:** Image MSE distribution. (a) Iterative reconstruction algorithm CT group. (b) CT group without the algorithm.

**Figure 10:** Comparison of the reconstructed images. (a) An ideal projection domain image and was relatively clear. (b) The noise projection domain image.

**Figure 11:** Comparison of the APACHE II scores between the two groups before and after treatment. ^∗^Significant difference compared with before treatment *P* < 0.01, ^#^after treatment, the difference between the observation group and the control group was significant, *P* < 0.01.

**Figure 12:** Comparison of severity factors in the patients of two groups. ^∗^Significant difference compared with before treatment, *P* < 0.01.

**Table 1:** Comparison of general data between the two groups.

	Control group	Observation group
Male	26	20
Female	24	30
Age	41.54 ± 2.18	43.54 ± 2.76
Overeating	22	19
Alcoholic	9	12
Hyperlipidemia	9	11
Biliary pancreatitis	8	10
*χ* ^2^	8.357	
*P*	0.256	

**Table 2:** Comparison of the survival rate between the two groups after treatment.

	Control group	Observation group
Survival (case)	45	50
Death (case)	5	1
Died of fungal sepsis (case)	2	0
Died of infective shock (case)	1	0
Died of renal failure (cases)	2	0
Survival rate (%)	90%	98%
*χ* ^2^	5.89	
*P*	0.002	

## Data Availability

The data used to support the findings of this study are available from the corresponding author upon request.
